# Effect of perioperative infusion of Dexmedetomidine combined with Sufentanil on quality of postoperative analgesia in patients undergoing laparoscopic nephrectomy: a CONSORT-prospective, randomized, controlled trial

This article has been retracted.

**DOI:** 10.1186/s12871-018-0608-3

**Published:** 2018-10-20

**Authors:** Fuxi Song, Chunmiao Ye, Feng Qi, Ping Zhang, Xuexiang Wang, Yanfeng Lü, Alejandro Fernandez-Escobar, Chao Zheng, Liang Li

**Affiliations:** 1 Department of Anaesthesiology, the Second Hospital of Shandong University, No. 247 Beiyuan Street, Jinan, 250033 China; 2 Department of Breast Surgery, the Second Hospital of Shandong University, No. 247 Beiyuan Street, Jinan, 250033 China; 3 Department of Anaesthesiology, Qilu Hospital of Shandong University, No. 107 Wenhua West Road, Jinan, 250012 China; 4 The Institute for Translational Medicine, the Second Hospital of Shandong University, No. 247 Beiyuan Street, Jinan, 250033 China; 5 Department of Anoproctology, the Second Hospital of Shandong University, No. 247 Beiyuan Street, Jinan, 250033 China; 6 Translational Research Program, University of Toronto, 27 King’s College Circle, Toronto, ON M5S 1A1 Canada

**Keywords:** Dexmedetomidine, Sufenanil, Postoperative analgesia, Flatus, Defecation

## Abstract

**Background:**

Postoperative pain is one of the most common symptoms after surgery, which brings physical discomfort to patients. In addition, it may cause a series of complications, and even affect the long-term quality of life. The purpose of this prospective, randomized, double-blinded, controlled trial is to investigate the efficacy and safety of dexmedetomidine combined with sufentanil to attenuate postoperative pain in patients after laparoscopic nephrectomy.

**Methods:**

Ninety patients undergoing laparoscopic nephrectomy were randomized into three groups: the control (sufentanil 0.02 μg/kg/h, Group C), sufentanil plus low dose of dexmedetomidine (0.02 μg/kg/h each, Group D1), and sufentanil plus high dose of dexmedetomidine (0.04 μg/kg/h, Group D2). The patient-controlled analgesia was programmed to deliver a bolus dose of 0.5 ml, followed by an infusion of 2 ml/h and a lockout time of 10 min. The primary goal was to calculate the cumulative amount of self-administered sufentanil; the secondary goals were to estimate pain intensity using the numerical rating scale (NRS), level of sedation, the first bowel movement, concerning adverse effects as well as duration of postoperative hospital stay.

**Results:**

The total consumption of sufentanil in group D1 and D2 were significantly lower than in group C during the first 8 h after surgery (*P* < 0.05), whereas there were no statistically significant differences (*P* > 0.05) between group D1 and D2. Compared with group C, the NRS scores at rest during first 8 h after surgery were significantly lower in group D1 (*P* < 0.05). The NRS scores, neither at rest nor with movement, show statistically significant differences between group D1 and D2 at each time point following surgery (*P* > 0.05). The time to first flatus was shorter in group D1 compared with the control group (*P* < 0.05). In addition, compared with group C, group D1 and D2 had a shorter time for first defecation (*P* < 0.05).

**Conclusions:**

Dexmedetomidine combined with sufentanil showed better postoperative analgesia without adverse effects, as well as facilitated bowel movements for patients undergoing laparoscopic nephrectomy.

**Trial registration:**

We registered this study in a Chinese Clinical Trial Registry (ChiCTR) centre on Dec 23 2015 and received the registration number: ChiCTR-IPR-15007628.

## Background

Postoperative pain is a common postoperative complication that can aggravate the body’s stress response. It can disturb the endocrine and immune function, as well as it is considered to be a risk factor for postoperative chronic pain. Meanwhile, severe postoperative pain will delay the recovery of patients after surgery, and even influence the quality of long-term survival [1–3]. Therefore, effective postoperative analgesia has a positive impacts on the recovery of patients following surgery. Ideal analgesia is defined as a measure that is easy to implement, effective, and has limited number of adverse effects. Postoperative patient-controlled analgesia (PCA) was introduced in the early 1980s. It is a delivery system that can be self-controlled by patients. Compared with traditional intramuscular injection of analgesia, PCA can be impactful as it alleviates postoperative pain, reduces drug consumption as well as it has less frequent postoperative complications [4].

Sufentanil is a selective μ - opioid receptor agonist that is characterized by its a fast onset, short duration of action and a strong analgesic effect (12-fold greater intrinsic potency than fentanyl) [5], has now become a common medication used in PCA. However, similar to other opioid drugs, sufentanil has significant side effects such as respiratory depression, nausea, vomiting and constipation [6]. In addition, it can potentially cause severe gastrointestinal adverse effects that may lead to dehydration, electrolyte imbalance, and a delay in enteral nutrition [7]. These will ultimately prolong hospital stay and increase the cost of hospitalization. Therefore, the ideal PCA should consist of a multimodal approach using a variety of drugs with different mechanisms of action that act synergistically, thereby reducing the opioid use and the incidence of side effects. Dexmedetomidine is a highly selective α 2-adrenergic receptor agonist with sedative and analgesic properties that has been associated with a relatively low incidence of adverse effects [8]. It has been widely used in intraoperative sedation, as well as in intravenous PCA as an adjuvant drug. However, there is still a paucity of evidence regarding the effect of dexmedetomidine in combination with sufentanil on postoperative outcomes for patients undergoing laparoscopic nephrectomy.

This prospective, randomized, double-blinded, controlled trial was designed to investigate whether a continuous application of dexmedetomidine and sufentanil for laparoscopic nephrectomy during perioperative period can decrease postoperative sufentanil consumption and pain intensity, as well as to validate the effectiveness and safety profile of this combined therapy.

## Methods

### Participants

This prospective, randomized, double-blinded, controlled trial was approved by the Institutional Medical Ethics Committee of Qilu Hospital of Shandong University on December 23, 2015 as it was in accordance with the current guidelines of the institution. This study was also registered at chictr.org (ChiCTR-IPR-15007628). Informed consent was obtained from all of the participants. We recruited patients who underwent laparoscopic nephrectomy under general anesthesia at Qilu Hospital from December 2015 to June 2016. This study was supported by the National Natural Science Foundation of China NSFC Grant No. 81702603, and the Key Project of the Natural Science Foundation of Shandong Province Grant No. ZR2014HZ004. The funders had no role in study design, data collection and analysis, decision to publish, or preparation of the manuscript.

Patients were selected to participate on the study based on the following inclusion criteria: age between 30 and 70 years; American Society of Anesthesiologists (ASA) physical status classification of I or II; intubated with an L-double-lumen endobronchial tube; received 48 h of intravenous PCA after surgery that was used with sufficient competence; agreed to cooperate and signed the informed consent.

Patients were excluded if they met the following criteria: body mass index (BMI) greater than 32 kg/m^2^; basal heart rate (HR) less than 55 beats/minute; history of ischemic heart disease within 6 months prior to this surgical procedure; second-degree or third-degree atrioventricular block; liver and kidney disfunction; history of chronic pain and long-term use of analgesic drugs (> 3 months); hypersensitivity to any of the test drugs; change in surgical approach was required (from laparoscopic to open surgery); failed to complete the data collection.

### Randomization and masking

After obtaining the informed consent, patients were allocated into three equal groups by an independent anesthetist who was blinded to the study, using a computer-generated randomization table. On the day of the surgery, this anesthetist prepared the intraoperative and postoperative intravenous PCA agents. During the postoperative period, the following outcomes were assessed: pain intensity using a numerical rating scale (NRS), both at rest and with movement; cumulative amount of self-administered sufentanil; level of sedation; concerning adverse effects such as nausea, vomiting, severe abdominal pain, abdominal distention, shivering, delirium, and serious respiratory depression.

### Anesthesia

All patients received atropine 0.5 mg by intramuscular injection in the ward, 30 min before entering the operating room (OR). After arriving to the OR, patients were randomly allocated into three groups by the anesthetist and a venous access was established on patients’ right upper limb by a nurse. All patients were continuously monitored using a 5-lead electrocardiogram, noninvasive blood pressure cuff, pulse oximetry saturation (SpO_2_), and end-tidal carbon dioxide (EtCO_2_) by an automated system (Philips IntelliVue MP50; Philips Company, Beijing, China). If these indicators appeared to be within the test standard, then a continuous infusion of the test drug would be immediately administered to the patient for a period of 10 min (groups D1 and D2 with 0.5 μg/kg DEX, group C with 0.9% NS). Propofol, sufentanil and rocuronium were given for anesthetic induction. After laryngeal mask airway (LMA) intubation, an arterial cannula was placed in the left radial artery. Anesthesia was maintained with sevoflurane (end-tidal concentration 1–2%), dexmedetomidine (0.9% NS in group C, 0.2 μg/kg/h in group D1 and 0.4 μg/kg/h in group D2), and rocuronium. The latter was given to provide a satisfactory level of muscle relaxation. Dexmedetomidine was stopped approximately 1 h prior to the end of surgery. If a fluctuation of more than 20% of the baseline level was evidenced in the mean arterial pressure (MAP), vasoactive drugs (serotonin 0.1–0.2 mg or nitroglycerin 50–100 μg) were used to maintain patients hemodynamically stable. In addition, if HR decreased to less than 50 beats/minute, atropine 0.5 mg was used. On the other hand, if HR increased to more than 100 beats/minute, esmolol 0.5 mg/kg was given to keep the patient stable. The EtCO_2_ was maintained at 28 to 38 mmHg. Thirty minutes before the end of surgery, palonosetron 0.25 mg was given to prevent post-operative nausea and vomiting (PONV). Neostigmine 0.04 mg/kg and atropine 0.02 mg/kg were administrated to revert neuromuscular blockade at the end of surgery. After endotracheal extubation, all patients were sent to the ward.

### Postoperative analgesia management

Before the surgery, all patients were instructed about the NRS, which ranged from 0 (no pain) to 10 (worst possible pain), as well as the how to use the intravenous PCA pump. The PCA was programmed to deliver a bolus dose of 0.5 ml followed by an infusion of 2 mL/h and a lockout time of 10 min. At the end of surgery, the PCA pump was started (Group C with sufentanil 0.02 μg/kg/h; group D1 with both sufentanil and DEX 0.02 μg/kg/h; group D2 with sufentanil 0.02 μg/kg/h and DEX 0.04 μg/kg/h). The goal of using the PCA was to maintain the NRS score less than 3 (at rest) in the first 48 h after surgery. If the NRS was greater than 3 (at rest), patients were given an additional bolus of sufentanil. If patients still reported pain or the NRS score was greater than 6 (at rest), supplemental rescue boluses of intravenous flurbiprofen axetil injection of 50 mg were administered. If the rescue analgesia was ineffective 30 min after administration, intravenous injection of tramadol (100 mg) was given.

### Outcome measures

The primary outcome measure was the cumulative amount of self-administered sufentanil. Furthermore, the secondary outcome measure were: pain intensity using NRS, both at rest and with movement; level of sedation (5-point scale: 0, patient is fully awake; 1, patient is drowsy/closed eyes; 2, patient is asleep/easily aroused with light tactile stimulation or a simple verbal command; 3, patient is asleep/arousable only by strong physical stimulation; and 4, patient is unarousable) [9], concerning adverse effects, the first bowel movement, and duration of postoperative hospital stay.

HR, MAP, and SpO_2_ were recorded at the following time points: 5 min after entering the OR (T0), 5 min after induction of anesthesia (T1), 5 min after establishment of pneumoperitoneum (T2), 1 h after establishment of pneumoperitoneum (T3), 5 min after stopping the sevoflurane (T4) and 5 min after extubation (T5). EtCO_2_ was recorded from T1 to T4. The cumulative amount of self-administered sufentanil and pain intensity were recorded at 1, 2, 4, 8, 16, 24 and 48 h after surgery; level of sedation was recorded at the time of tracheal extubation, 1, 2 and 4 h after surgery; The total number of rescue analgesia and the postoperative adverse effects (nausea and vomiting, severe abdominal pain, abdominal distention, drowsiness, shivering, delirium, and serious respiratory depression) were also recorded at the end of the study.

### Statistical analysis

Statistical analysis was performed with SPSS for Windows Version 21.0 (SPSS Inc. Chicago, IL). We used the Kolmogorov - Smirnov test to assess distribution of the variables. Homogeneity of variance was compared among the three groups by Levene tests. Normally distributed data were expressed as mean standard deviation, skewed data distribution was expressed using median, and categorical data were expressed as frequency (n) and percentage (%). Parameters like age, weight, operation time, anesthesia time, bowel movement recovery time, dosage of sufentanil and MAP, HR, EtCO_2_, SpO_2_ at different time points among the groups were compared using 2-way analysis of variance (ANOVA). Multiple comparisons were performed using the LSD post hoc test. NRS and level of sedation were compared among the three groups with Mann-Whitney test, and categorical variables were analyzed using x^2^ test. All data with Probability (P) values < 0.05 were considered statistically significant.

## Results

A total of 112 patients undergoing laparoscopic nephrectomy were screened between December 2015 and June 2016, of which 17 were excluded because they either did not meet the inclusion criteria or refused to participate in the trial. The remaining 95 patients were randomly allocated into three groups. Two patients were eliminated due to conversions to open nephrectomy (one from group D1 and one from group D2), and one patient cancelled the surgery (from group D2). Another two patients were excluded after surgery due to incomplete clinical data (one from group C, one from group D1). (Fig. 1).

**Fig. 1:** Patient enrolment flow diagram. This illustrates the flow of all patients screened, excluded, and randomized

### Demographic data and surgery/anesthesia related information

Baseline characteristics and demographics of patients were compared among the three groups (Table 1). No statistically significant differences were found in sex, age, height, body weight, BMI and ASA grade (*P* > 0.05; Table 1). Hypertension was the most frequent type of basic disease as it affected 36.67%, 36.67%, 43.33% of group C, D1 and D2, respectively; there were no statistically significant differences in type of underlying disease and surgeries. The intraoperative data and recovery time among the three groups appeared to have no statistically significant differences (*P* > 0.05; Table 1). Changes in MAP, HR, EtCO_2_ and SpO_2_ among the three groups showed no statistical significance (*P* > 0.05; Fig. 2).

**Table 1:** Clinical Characteristics of Patients in Group C, D1 and D2

	Group O(*n* = 30)	Group D1(*n* = 30)	Group D2(*n* = 30)	*P* value
Sex, F/M,n	10(33.33%)/20(66.67%)	5(16.67%)/25(83.33%)	8(26.67%)/22(73.33%)	0.330
Age, years	51.50 ± 12.06	50.27 ± 10.06	50.94 ± 9.91	0.890
BMI, kg/m^2^	26.24 ± 2.84	26.09 ± 1.46	25.83 ± 2.23	0.785
basic disease(hypertension /DM/CHD), n(%)	7(23.33%)/3(10.00%)/1 (3.33%)	9(30.00%)/2(6.67%)/ 0(0%)	11(36.67%)/2(6.67%)/0(0%)	0.840
Type of surgery (radical/ partial), n(%)	14(46.67%)/16 (53.33%)	16(53.33%)/14(46.67%)	14(46.67%)/16(53.33%)	0.850
ASA I/II, n(%)	4(13.33%)/26(86.67%)	2(6.67%)/28(93.33%)	1(3.33%)/29(96.67%)	0.338
Duration of anaesthesia, min	152.50 ± 63.63	149.67 ± 53.38	143.67 ± 57.63	0.836
Duration of surgery, min	134.00 ± 58.63	136.33 ± 53.22	128.83 ± 57.11	0.870
Duration of analgesia, min	20.67 ± 12.98	15.50 ± 5.78	17.90 ± 6.32	0.089
2%propofol, ml	14.43 ± 1.85	14.73 ± 1.25	14.13 ± 1.36	0.311
Rocuronium, mg/h	35.73 ± 6.55	36.26 ± 6.37	37.52 ± 6.55	0.552
Sufentanil,μg	34.50 ± 10.45	30.67 ± 1.72	31.50 ± 3.97	0.063
Number of using vasoactive agent, n (%)	17 (56.67%)	14 (46.67%)	13 (43.33%)	0.219
Postoperative stay in hospital, d	9.40 ± 1.10	8.90 ± 0.85	9.20 ± 0.83	0.243

Variables presented as mean SD or number of patients n (%). None showed any statistical significance (*P* > 0.05)

*ASA* American Society of Anesthesiologists, *BMI* body mass index, *CHD* coronary heart disease, *DM* diabetes mellitus, *SD* standard deviation

**Fig. 2:** Changes in MAP, HR, EtCO_2_ and SpO_2_ among the three groups. Continuous variables presented as mean standard deviation. None showed any statistical significance (*P* > 0.05). (T0, 5 min after entering the OR; T1, 5 min after induction of anesthesia; T2, 5 min after establishment of pneumoperitoneum; T3, 1 h after establishment of pneumoperitoneum; T4, 5 min after stop sevoflurane; T5, 5 min after extubation), HR = heart rate, MAP = mean arterial pressure, SpO_2_ = pulse oxygen saturation, EtCO_2_ = end-tidal carbon dioxide partial pressure, OR = operating room

### Postoperative outcome

The total consumption of sufentanil was lower in group D1 and D2 compared with group C at 1, 2, 4 and 8 h after surgery (*P* < 0.05; Table 2), whereas the total dosage of sufentanil had no statistically significant differences between group D1 and D2 at any time point after surgery (*P* > 0.05; Table 2). In addition, patients that needed additional self-administered sufentanil within 48 h after surgery in group D1 (10 cases) and group D2 (11 cases) were significantly lower than group C (20 cases) (*P* < 0.05 Table 2). The NRS score at rest during the first 8 h after surgery was significantly lower in group D1 compared with group C (*P* = 0.012). In addition, the NRS scores with movement at 1, 2, 4, 8, 24 and 48 h after surgery were significantly lower in both group D1 and D2 (*P* < 0.05; Fig. 3). The NRS scores both at rest and with movement showed no statistically significant differences between group D1 and D2 at each time point after surgery (*P* > 0.05; Fig. 3). No patients required rescue analgesia in any of the three groups, 48 h after surgery (Table 2).

**Table 2:** Total Dosage of Sufentanil in Group C, D1 and D2

	Time point	Group C(*n* = 30)	Group D1(*n* = 30)	Group D2(*n* = 30)	*P* values(P_c and D1_, P_c and D2_, P_D1 and D2_)
Concentration of sufentanil, μg/ml		0.77 ± 0.11	0.76 ± 0.06	0.72 ± 0.06	0.163(0.552/ 0.063/ 0.200)
Dosage of sufentanil, ml	1 h	2.28 ± 0.41	2.00 ± 0.00	2.05 ± 0.15	0.003(0.001**/0.007**/0.531)
	2 h	4.27 ± 0.41	4.05 ± 0.15	4.12 ± 0.29	0.013(0.011*/0.011*/1.000)
	4 h	8.40 ± 0.50	8.10 ± 0.30	8.13 ± 0.22	0.020(0.012*/0.020*/0.829)
	8 h	16.48 ± 0.57	16.16 ± 0.46	16.17 ± 0.34	0.058(0.032*/0.047*/0.866)
	24 h	48.55 ± 0.69	48.25 ± 0.77	48.17 ± 0.34	0.143(0.135/ 0.063/ 0.706)
	48 h	96.55 ± 0.69	96.30 ± 0.92	96.17 ± 0.35	0.227(0.258/ 0.092/ 0.570)
Needed additional self- administered sufentanil, n(%)	48 h	20(66.67%)	10(33.33%)	11(36.67%)	0.051(0.030*/0.039*/0.930)
Needed rescue analgesia, n(%)	48 h	0 (0%)	0 (0%)	0 (0%)	1.000

Variables presented as mean SD or number of patients n (%). The total consumption of sufentanil were significantly lower in group D1 and D2 than group C at 1, 2, 4 and 8 h after surgery. Patients that needed additional self-administered sufentanil within 48 h after surgery in group D1 and group D2 were significantly lower than in group C. (* meant P < 0.05 compared with Group C, **meant P < 0.01 compared with Group C)

No patients required rescue analgesia in all the three groups 48 h after surgery

**Fig. 3:** Pain score (NRS) during 48 h after surgery in group C, D1, and D2. Variables presented as mean standard deviation. The NRS score at rest during the first 8 h after surgery was significantly lower in group D1 compared with group C (*P* = 0.012). The NRS scores with movement at 1, 2, 4, 8, 24 and 48 h after surgery were significantly lower compared group D1 with group C (*P* = < 0.001, < 0.001, 0.010, 0.032, 0.024, 0.006, respectively). At the same time, compared with group C, group D2 also show significantly lower NRS scores with movement at 1, 2, 4, 8, 24 and 48 h (*P* = < 0.001, 0.002, 0.005, 0.027, 0.001, 0.028, respectively). (*meant *P* < 0.05 compared group D1 with group C; # meant *P* < 0.05 compared group D2 with group C). NRS = numerical rating scale

Level of sedation was monitored within the first 4 h post-surgery. The findings were summarized in Table 3. Between the three groups, there were no statistically significant differences among the patients at any time point after surgery (*P* > 0.05; Table 3). Patients in group D2 had more drowsiness than patients in group D1 and C (*P* < 0.05; Table 4). Other adverse effects had no statistically significant differences among the three groups (*P* > 0.05; Table 4).

**Table 3:** Level of sedation in Group C, D1 and D2

	Time point	Group O(*n* = 30)	Group D1(*n* = 30)	Group D2(*n* = 30)	*P* values(P_c and D1_, P_c and D2_, P_D1 and D2_)
level of sedation (0/1/2/3), n	extubation	2 (1–3)	2 (1–2)	2(1–2)	0.542/0.737/ 0.755
	1 h	1 (0–2)	1 (0–1)	1 (0–2)	0.060/ 0.630/ 0.007
	2 h	0 (0–2)	0 (0–1)	1 (0–2)	0.450/ 0.771/ 0.287
	4 h	0 (0–1)	0 (0–1)	0 (0–1)	0.080/ 0.218/ 0.553

Variables presented as median (interquartile range) or number of patients, n

**Table 4:** Adverse reactions after Surgery in Group C, D1 and D2

	Group O(*n* = 30)	Group D1(*n* = 30)	Group D2(*n* = 30)	*P* values
Nausea and Vomiting	7 (43.33%)	5(30%)	5 (26.67%)	0.495
Severe abdominal pain and distention	4 (13.33%)	5 (16.67%)	4 (20%)	0.787
Drowsiness	1 (0%)	2 (6.67%)	7 (23.33%)	0.031^*^
Delirium	0 (0%)	0 (0%)	0 (0%)	1.000
Shivering	1 (3.33%)	1 (6.67%)	0 (0%)	0.537
serious respiratory depression	0 (0%)	0 (0%)	0 (0%)	1.000

Variables presented as number of patients, n (%) *meant P < 0.05

The first flatus and defecation time after surgery of patients in group D1 and D2 were significantly shorter than group C (*P* < 0.05, Fig. 4). Moreover, the difference between D1 and D2 in terms of postoperative bowel movement had no statistical significance (*P* > 0.05, Fig. 4).

**Fig. 4:** Bowel movement recovery after surgery among the three groups. Variables presented as mean standard deviation.* meant *P* < 0.05 compared group D1 with group C; # meant *P* < 0.05 compared group D2 with group C

## Discussion

This prospective, randomized, double-blinded, controlled trial showed that using dexmedetomidine combined with sufentanil in patients could decrease the total dosage of sufentanil and improve postoperative analgesia during the first 8 and 48 h after surgery, respectively. In addition, the first flatus and defecation time after surgery in patients of group D1 and D2 were evidently shorter than group C. Patients that were administered a high dose of dexmedetomidine (0.04  μg/kg/h) experienced more drowsiness compared to the participants in the other two groups.

The beneficial effects of dexmedetomidine for postoperative analgesia have been reported in many reviews [10–12]. In some clinical studies, the combination of dexmedetomidine and opioids for postoperative intravenous PCA could significantly reduce the consumption of opioids in more than 24 h after surgery [3, 13, 14]. In contrast to those reports, in our study, using dexmedetomidine demonstrated to lessen the required dosage of sufentanil, but the degree of reduction was not clear compared with the total uses of sufentanil. The pain scores (NRS) at rest had no statistically significant differences except during the first 8 h after surgery (NRS at 8 h after surgery in group D1 was evidently lower than in group C), while the pain scores (NRS) with movement in group D1 and D2 were clearly lower than in group C at any time point within 48 h after surgery. The reasons to explain these differences may be complex. Firstly, opioid and α 2-adrenergic receptor agonists are both potent analgesic drugs that can work synergistically when co-administered. Some studies have also shown that the combination of α 2-adrenergic receptor agonists and opioid agonists in sub-analgesic dose can also achieve an effective analgesic effect [15, 16]. This synergistic interaction takes effect in the spinal cord due to the presence of the receptors that mediate these interactions and cause downstream signaling events that ultimately enable the synergy to occur [17]. Secondly, compared with traditional open nephrectomy, laparoscopic nephrectomy has benefits of a smaller incision and less postoperative pain [18, 19]. In our study, the administration of sufentanil 0.2 μg/kg/h was sufficient to satisfy the needs of postoperative analgesia in patients undergoing laparoscopic nephrectomy; only a few patients required additional self-administered doses of sufentanil. The level of pain in patients at rest demonstrated no statistically significant different among the three groups. Therefore, infusion of dexmedetomidine could only slightly decrease the amount of sufentanil. In the meantime, the pain scores (NRS) in the three groups showed no statistically significant differences. Further research is necessary to explain the reasons for the differences observed with regards to the effect of dexmedetomidine on pain between rest and movement.

This pilot study showed that dexmedetomidine could increase the incidence of drowsiness that is easily arousable and does not cause severe respiratory depression; this is consistent with its sedative effect [8, 20]. According to Song et al. [21], dexmedetomidine added to an opioid-based analgesic regimen could prevent PONV in highly susceptible patients. However, in our study, there appeared to be no differences in the occurrence of PONV between the three groups. This was mainly prevented by an adequate bowel preparation and antiemetic drug application during the perioperative period. Additionally, laparoscopic nephrectomy had less stimulation of gastrointestinal tract compared to an open nephrectomy. All of these contributed to a low incidence of PONV among the three groups. Talke et al. [22] reported that bradycardia and hypotension are the most common side effects of dexmedetomidine. However, in our study, no patients were found to have bradycardia or hypotension. It may have been primarily due to the criteria of patient enrollment that was adopted in our study (patients with a history of ischemic heart disease 6 months prior to this event or history of second-degree or third-degree atrioventricular blocks were excluded). In addition, age, PCA settings, monitoring protocol and type of surgery could have also influenced the results.

In this prospective study, we also found that the combination of dexmedetomidine with opioids improved the recovery of bowel movement after surgery which is in accordance with the previous report by Jin et al. [23]. Sympathetic activation has been demonstrated that it is related to the occurrence and development of postoperative ileus [24–26]. Dexmedetomidine can inhibit the excessive activation of the sympathetic nervous system [27], therefore causing a decreased inhibitory effect in the gastrointestinal tract. In addition, the inhibitory effect of sympathetic nervous system can decrease acetylcholine release, which is crucial for the activation of the enteric nervous system. Opioids such as sufentanil can induced bowel dysfunction [28], while the use of dexmedetomidine reduces the dosage of sufentanil used after surgery, thereby reducing the inhibition caused by it.

Although some studies have proved that dexmedetomidine can decrease the incidence of postoperative delirium [29, 30], there is no sufficient evidence in our trial to support this argument. However, delirium usually occurs in elderly patients or patients with prolonged-operative time, while in our study, all surgical procedures had a short operative time, therefore decreasing the likelihood of finding delirium in our patients. In addition, the incidence of other adverse effects can also be attributed to a similar reason.

Some limitations exist in our study. First of all, instead of monitoring the depth of anesthesia by BIS value, we maintained the depth of anesthesia by adjusting the sevoflurane end-tidal concentration, but it could not accurately reflect the depth of anesthesia. Secondly, dexmedetomidine was administered at a rate of 0.5  μg/kg for 10  minutes before the induction of anesthesia and then at a rate of 0.2 to 0.4 μg/kg/h during the operation. We did not measure the serum concentration of dexmedetomidine at any time point, so we could not determine the effects of the plasma concentrations of dexmedetomidine on intraoperative hemodynamics. Finally, laparoscopic nephrectomy has two different surgical approaches, intra-abdominal and retroperitoneal. Therefore, different surgical techniques could have influenced the postoperative analgesia and bowel movement recovery, but we did not take this into account. To further investigate this effect on postoperative outcomes, more studies are required.

## Conclusions

In conclusion, we found that combination of sufentanil and dexmedetomidine (0.02–0.04  μg/kg/h) was associated with better analgesic effect, and faster recovery of bowel movement without additional severe adverse effects in patients after laparoscopic nephrectomy compared with sufentanil alone. To decrease the incidence of drowsiness, we suggested using low dose of dexmedetomidine (0.02  μg/kg/h) instead of high dose of dexmedetomidine (0.04  μg/kg/h). More studies are still required to determine the optimal dose of dexmedetomidine for improving postoperative analgesia in patients undergoing other types of surgeries.

## Abbreviations

ASA: American Society of Anesthesiologists
BMI: Body mass index
CHD: Coronary heart disease
DM: Diabetes mellitus
EtCO_2_: End-tidal carbon dioxide partial pressure
HR: Heart rate
LMA: Laryngeal mask airway
MAP: Mean arterial pressure
NRS: Numerical rating scale
NS: Normal saline
OR: Operating room
PCA: Patient-controlled analgesia
PONV: Postoperative nausea and vomiting
SpO_2_: Pulse oxygen saturation
